# Keratoconus Classification with Convolutional Neural Networks Using Segmentation and Index Quantification of Eye Topography Images by Particle Swarm Optimisation

This article has been retracted.

**DOI:** 10.1155/2022/8119685

**Published:** 2022-03-22

**Authors:** Subramanian P., Ramesh G. P.

**Affiliations:** Department of Electronics and Communication Engineering, St Peter's Institute of Higher Education and Research, Chennai, India

## Abstract

In keratoconus, the cornea assumes a conical shape due to its thinning and protrusion. Early detection of keratoconus is vital in preventing vision loss or costly repairs. In corneal topography maps, curvature and steepness can be distinguished by the colour scales, with warm colours representing curved steep areas and cold colours representing flat areas. With the advent of machine learning algorithms like convolutional neural networks (CNN), the identification and classification of keratoconus from these topography maps have been made faster and more accurate. The classification and grading of keratoconus depend on the colour scales used. Artefacts and minimal variations in the corneal shape, in mild or developing keratoconus, are not represented clearly in the image gradients. Segmentation of the maps needs to be carried out for identifying the severity of the keratoconus as well as for identifying the changes in the severity. In this paper, we are considering the use of particle swarm optimisation and its modifications for segmenting the topography image. Pretrained CNN models are then trained with the dataset and tested. Results show that the performance of the system in terms of accuracy is 95.9% compared to 93%, 95.3%, and 84% available in the literature for a 3-class classification that involved mild keratoconus or forme fruste keratoconus.

## 1. Introduction

Keratoconus refers to the condition of the eye wherein the cornea assumes a cone shape rather than the normal dome shape [1]. Keratoconus can affect any one eye (unilateral) or both eyes (bilateral) and can vary in the degree of progression between the two eyes (asymmetric) [2]. Keratoconus may lead to loss of vision in extreme cases or might require corrective procedures including lenses. Keratoconus in the advanced stage is clearly visible and detectable in the form of Munson's sign, Vogt's striae, Fleischer's Ring, etc. [3]. But the early signs of keratoconus are difficult to identify. Tools like video keratoscope have been used to identify the early signs using corneal topography images. Several topography indices have been used to identify and classify the keratoconus. But with the large number of indices, it is difficult to do the identification process manually. Computerised diagnosis also requires selection of indices that are more relevant, to reduce the computing time and errors. Dimensionality reduction techniques have been employed to some extent to reduce the number of parameters or indices. The advent of machine learning and deep learning architectures has helped in the diagnosis of keratoconus. Convolutional neural networks have been used extensively in the diagnosis of medical conditions including breast cancer diagnosis, brain tumour segmentation, Alzheimer's disease, Parkinson's disease, lung diseases, diabetic retinopathy, and keratoconus. In this paper, we consider applying segmentation of the topography images for segmentation and identifying the indices and then use convolutional neural networks for the diagnosis and classification of keratoconus. The rest of the paper has the following sections. In Related Works, we discuss on the prevailing CNN architectures and optimisation techniques available in the literature for medical diagnosis with emphasis on applications for keratoconus diagnosis and classification. In Proposed Method, we discuss on the dataset, network architecture, and optimisation employed. In Results and Discussion, we discuss and compare the results obtained with different architectures and optmisation"with"optimisation methods. Conclusion includes the conclusion statement and future directions for the work.

## 2. Related Works

Machine learning has been used extensively in the diagnosis and classification of keratoconus. A brief discussion on the application of machine learning for keratoconus identification and classification, available in the literature, is presented here.  Table 1 lists the different networks used for classification and their performance.

Accardo and Pensiero [4] have used a three-layered neural network with backpropagation training for classification as normal, keratoconus, and others. Different architectures were considered by varying the number of input, hidden, and output layers. Maps from single eye and both eyes of the same patient have been considered for classification. Different combinations of layer sizes and learning rate parameters have also been considered resulting in varying global sensitivities. The authors have achieved global sensitivity ranging from 81.7 to 94.1 and global accuracy of 92.9 to 96.4. The results vary with consideration of the single or both eyes. With single eye, the accuracy level decreases. Also, the network was not able to classify subclinical or forme fruste keratoconus.

Souza et al. [5] have considered only one eye of each patient. Eleven attributes are shortlisted from Orbscan II and are applied as input parameters for different algorithms, namely, radial basis function neural network (RBFNN), multilayer perceptron (MLP), and support vector machine (SVM). The parameters used included anterior and posterior best fit spheres, maximum and minimum simulated keratometry, maximum anterior and posterior elevation, 5 mm irregularity, thinnest point, and central corneal power. The system provides detection of keratoconus but does not provide classification of stages of keratoconus. Different combinations of attributes need to be considered apart from the eleven attributes considered, and data from both eyes of the patient can be considered.

MLP, RBFNN, SVM, and decision tree (DT) are employed by Toutounchian et al. [6] with direct features from Pentacam and features derived from topographical images. The attributes directly obtained from Pentacam are corneal thickness, anterior and posterior best fit spheres, progression index, sagittal curvature, tangential curvature, relative pachymetry, corneal thickness spatial profile, and age. The second group of features consists of Randleman score system, Ambrosia score system, and symmetry in sagittal map. Though better accuracy for distinguishing between normal and keratoconus eyes has been obtained, the accuracy level decreases when suspect to keratoconus is involved.

Arbelaez [7] has classified the eyes as abnormal, keratoconus, subclinical keratoconus, and normal using support vector machine (SVM). There were four groups of eyes, based on clinical diagnosis, namely, clinically diagnosed keratoconus, clinically diagnosed subkeratoconus, eyes undergone refractive surgery, and normal eyes. The precision of classification increases in the distinction between normal and subclinical cases, when posterior corneal surface data are included. The accuracy levels are the least with respect to the subclinical keratoconus in both cases.

Hidalgo et al. [8] have used support vector machine (SVM) with linear kernel that employs dimensionality reduction. The eyes are fist classified by specialists into normal, astigmatism, postrefractive surgery (PRS), forme fruste (FF), and keratoconus. Pentacam provides around 1000 parameters which include correlated variables raising the need for reduction to reduce computation. Correlation-based hierarchical clustering is employed resulting in a dendrogram followed by selection of one variable from each branch. This resulted in the selection of 22 parameters. The classification performance indicates that the performance is less for forme fruste keratoconus classification, with the sensitivity as low as 37.3%, compared to others.

Lavric and Popa [9] used a convolutional neural network (CNN) for extracting and learning the features of a keratoconus eye. Topographic maps with colour scales are used for analysis. Here, warm colours are used to represent curved/steep areas and mild colours are sued for flat areas. SyntEyes KTC model has been used to generate input data to overcome the difficulty in obtaining real data from patients. The accuracy obtained by Lavric is in the range of 99.33%, and this can be used as a screening mechanism by ophthalmologist. The performance of the system depends on the image steps used, with smaller steps increasing the sensitivity and larger steps resulting in missing the mild cases of keratoconus.

Santos et al. [10] have employed a customized fully convolutional neural network, CorneaNet, for early detection of keratoconus. The network is used for segmentation of OCT images. The thickness maps of full cornea, Bowman layer, epithelial layer, and stroma are used, and the segmentation speed considerably improved with the usage of the CorneaNet. In cornea with keratoconus, the thin zone could be detected and used for early detection of keratoconus with 99.5% accuracy.

Kamiya et al. [11] have obtained improved diagnostic accuracy by using deep learning on six colour-coded maps, namely, anterior elevation map, anterior curvature map, posterior elevation map, posterior curvature map, refractive power map, and pachymetry map. Six neural networks were trained for classification into 4 grades by taking into the average of the six outputs. Comparison of accuracy of the classification between normal and keratoconus eyes shows that the accuracy improves when the six maps were used when compared with the usage of the individual maps.

Lavric et al. [12] have integrated the data generated in the SyntEyes algorithm with anterior and posterior keratometry along with pachymetry. The anterior keratometry is added with the input CNN. The network provides the classification as normal and keratoconus eyes.

Shi et al. [13] have used neural network-based machine learning for classification of eyes into normal, keratoconus, and subclinical keratoconus eyes. Combined features from Scheimpflug-based camera and ultrahigh-resolution optical coherence tomography (UHR-OCT) provided better discrimination between the three classes than the features obtained from a single instrument. The UHR-OCT provides better discrimination between the subclinical and clinical keratoconus.

Kuo et al. [14] have used three well-known CNN models, namely, VGG16, InceptionV3, and ResNet152, for detecting the pattern differences between normal and keratoconus eyes. The networks provided accuracy of 0.931 to 0.958. It has been observed that the results depend on the patterns and not on the colour scales used and hence can be used across different platforms. Also, the classification of subclinical cases was less satisfactory compared to the keratoconus cases.

Lavric et al. [15] have compared the performances of 25 different models in machine learning with an accuracy ranging from 62% to 94.0%. The best performance of 94% has been observed in a support vector machine (SVM) that used eight corneal parameters which were selected using feature selection.

Thulasidas and Teotia [16] have observed that the usage of pachymetric progression index and the BAD-D value resulted in improved detection of subclinical keratoconus when compared to the use of other Pentacam parameters as inputs. It is also observed that a combination of data results in improved detection of subclinical keratoconus rather than that of a single parameter.

Hallet et al. [17] employed a multilayer perceptron and variational autoencoder for classification of keratoconus and normal eyes. The unsupervised variational autoencoder gives better results with 80% accuracy when compared with the supervised multilayer perceptron with 73% accuracy.

Daud et al. [18] used a smart device to capture posterior and anterior segment eye images, which were segmented to extract the geometric features using automated modified active contour model and the semiautomated spline function. Feature selection is carried out using infinite latent feature selection (ILFS).

Mahmoud and Mengash [19] have presented the 3-dimensional construction of corneal images from the 2-dimensional front and lateral images of the eye for detection of keratoconus and its stages. The convolutional neural network used for feature extraction uses the constructed 3-dimensional image. The accuracy of diagnosis obtained is 97.8% with a sensitivity of 98.45% and specificity of 96.0%.

Feng et al. [20] have proposed a customized CNN, KerNet, for detecting keratoconus and subclinical keratoconus, from the Pentacam data. The data selected from Pentacam included the curvature of the front and back surfaces, elevation of the front and back surfaces, and the pachymetry data in the form of numerical matrices. The network proposed, KerNet, uses multilevel fusion architecture. The proposed network improves the accuracy of the detection of keratoconus by 1% and subclinical keratoconus by 4%.

Lavric et al. [21] have employed support vector machine to classify the different severity levels of the keratoconus apart from the regular classification of normal, subclinical, and keratoconus. Starting with 2-class classification of healthy and keratoconus eyes with the highest area under curve (AUC) of 0.99, the work has been extended to a 3-class classification of normal, forme fruste, and keratoconus eyes with an AUC of 0.96. Further extension to a five-class classification as normal, forme fruste, stage II, stage III, and stage IV yielded an AUC of 0.88.

Zaki et al. [22] used lateral segment photographed images (LSPI) which were extracted from videos of patients taken sideways with a smartphone camera. VGGNet 16 model is used for the classification achieving 95.75% accuracy, 92.25% sensitivity, and 99.25% specificity.

## 3. Proposed Method

The advent of machine learning has greatly helped in the identification of keratoconus as can be seen in the articles available in the literature. Of particular concern is the diagnosis of the mild keratoconus or forme fruste keratoconus. Diagnosis based on the measured parameters, running into thousands, involves dimensionality issues, while the selection of particular parameters alone involves accuracy issues. Diagnosis and classification of keratoconus from eye topography images are developing due to the computing power of deep networks in case of image data. The topography images are fraught with the problems involving artefacts and colour scales used. The colour scales used vary the accuracy of the results since the corneal elevation and the indices are dependent on the colour scales used in the topography images. Collection of datasets for keratoconus has been difficult due to the less prevalence of the disease, and there is no availability of a standard dataset as in cases of other image datasets. Hence, the SyntEye KTC model (Rozema et al.) has been used to generate the dataset that is to be used for the training of the CNN. The dataset consists of topography images of healthy normal eyes, developing keratoconus eyes, and keratoconus eyes.  Figure 1 shows the methodology and the steps involved in the proposed system.

Particle swarm optimisation techniques including PSO, DPSO, and FPSO are used for the segmentation and linearisation of the indices of topography images for better results. The optimised dataset is divided into training set and testing set. The training set is used to train the CNN and the testing is done using the testing set. VGG16 a pretrained CNN model is then used for transfer learning (Figure 2). The results are compared with both optimised and unoptimised datasets.

Particle swarm optimisation (PSO) is easy to implement and faster with few parameters to be adjusted. The particle swarm optimisation has the ability to converge faster to a solution and also involves only basic mathematical operators and not derivatives which are hard to implement. Particle swarm optimisation consists of a swarm or group of particles with each particle representing a potential solution. Here, the intensity each particle *N*_*i*_ is compared with intensity *L*_*i*_ of each particle of the input image. If *L*_*i*_ is greater than *N*_*i*_, then a variable *a* is incremented by 1 and the intensity is added to another variable *b*. Similarly, if *L*_*i*_ is less than *N*_*i*_, then a variable *c* is incremented by 1 and the intensity is added to the variable *d*. The fitness function to be evaluated is now given by fitness(*i*) = *c*_∗_ *a*_∗_ ((*d*/*c*) − (*b*/*a*))^2^. In DPSO, the search space is defined by *N* = {*Ni*}. The objective function *L* for mapping *N* is represented by NL➔ *J* = {*Ji*}. The neighbourhood elements represent search space *N* separated by distance “*d*”. The search space *N* has finite states and discrete function *L*. The DPSO can be used when the particle velocity and position are defined.

The fractional order PSO (FPSO) is given by equation (1).

(1) $$\begin{array}{c} \nabla^{v}x\left(k\right)=\overset{k}{\underset{j=0}{\sum }}\;{\left(-1\right)}^{j}\left(\begin{array}{c} v\\ j \end{array}\right)x\left(k-j\right), \end{array}$$

where the fractional order *v* is represented by equation (2).

(2) $$\begin{array}{c} \left(\begin{array}{c} v\\ j \end{array}\right)=\left\{\begin{array}{cc} 1, & \text{ for }j=0,\\ \frac{v\left(v-1\right)\cdots \left(v-j+1\right)}{j!}, & \text{ for }j>0. \end{array}\right. \end{array}$$

Compared to PSO, the FPSO has different topology and initial velocity of particle and different acceleration rate of particles. The velocity of particle by order difference is represented by

(3) $$\begin{array}{c} \begin{array}{c} V_{i}\left(k+1\right)=\left(w\left(k\right)+\alpha -1\right)V_{i}\left(k\right)+c_{1}r_{1}\left(P_{i}\left(k\right)-x_{i}\left(k\right)\right)+\\ c_{2}r_{2}\left(P_{g}\left(k\right)-x_{i}\left(k\right)\right)+\overset{L}{\underset{p=1}{\sum }}\;C_{p}V_{i}\left(k-p\right) \end{array}, \end{array}$$

where *C*_*p*_ represents convergence in to 0, *V*_*i*_ represents velocity of *i*th particle, *k* represents difference of velocity for particles, and *P* = 1,2,3 to *k*.

The FPSO through multiple velocity and acceleration for different particles determines the regions with thin cornea in topography images.

## 4. Results and Discussion

The SyntEye KTC model is used to generate topography images of normal, subclinical keratoconus, and keratoconus eyes. 500 images were generated for each category. The generated images are then subject to PSO, DPSO, and FPSO for removing the artefacts as well as for delineating the corneal images for improving the number of indices. The CNN model used is the GoogLeNet model. Transfer learning approach is used for the classification problem, wherein the classification is of three categories, namely, normal, subclinical keratoconus, and keratoconus. The network is trained with 900 images comprising 300 from each category and then tested with the remaining 600 images. The process is repeated for the optimised images, namely, PSO, DPSO, and FPSO, and the results are compared in terms of accuracy, specificity, and sensitivity.

Accuracy defines the correctness of the model or the ratio of correct classification to the total number of inputs. It is given by

(4) $$\begin{array}{c} \text{Accuracy}=\frac{\left(\text{TP}+\text{TN}\right)}{\text{Total Number of Eyes}}. \end{array}$$

Specificity represents the model's ability to correctly identify as not belonging to a particular class, i.e., the true negative rate, and is given by

(5) $$\begin{array}{c} \text{Specificity}=\frac{\text{TN}}{\left(\text{TP}+\text{FN}\right)}. \end{array}$$

Sensitivity represents the model's ability to correctly identify an input as belonging to a particular class, i.e., the true positive rate, and is given by

(6) $$\begin{array}{c} \text{Sensitivity}=\frac{\text{TP}}{\left(\text{TP}+\text{FN}\right)}. \end{array}$$

Here, TP represents the true positive which is the number of cases identified correctly as belonging to a particular class. TN represents true negative which is the number of cases identified correctly as not belonging to a particular class. FP represents false positive which is the number of cases wrongly identified as belonging to a particular class, and FN represents the false negative which is the number of cases wrongly identified as not belonging a particular class.

Results obtained have accuracy levels of 94.3%, 95.3%, and 95.9% for the three variations of optimisation techniques used. The specificity values obtained are 95.8%, 96.6%, and 97%. The sensitivity levels obtained are 91.8%, 93.2%, and 94.1%. Tables 2, 3, and 4 give the confusion matrices for different optimisation techniques.  Figure 3 depicts the performance in terms of accuracy, specificity, and sensitivity of the systems with particle swarm optimisation of the dataset.  Figure 4 depicts the performance in terms of accuracy, specificity, and sensitivity of the system with DPSO-optimised dataset.  Figure 5 shows the accuracy, specificity, and sensitivity of the system using FPSO-optimised dataset particle swarm optimisation of the dataset.  Table 5 compares the performance of our proposed system with existing systems for a 3-class keratoconus classification. We can observe that the classification parameters are better for the case wherein the input topography images are optimised with FPSO.

## 5. Conclusion

Identification and classification of keratoconus have improved with the advent of the machine learning techniques. CNN is more prevalently used for the classification of corneal topography images. The availability of large datasets of corneal topography images has been an issue and is solved to an extent by synthesis of topography images combined data augmentation methods. The classification accuracy levels achieved, though high for two classifications as normal and keratoconus, decrease when a third class of mild keratoconus is involved. The present work was aimed at improving the classification accuracy of the mild or forme fruste keratoconus. The improvisation comes in terms of the optimisation techniques applied for segmenting the corneal topography images. The present research work utilized PSO, discrete PSO, and fractional PSO performed in initial set of process before using the topology images for testing and training the CNN. Results showed improved performance in terms of accuracy, sensitivity, and specificity when optimisation is done and also with the results available in the literature with three class classifications of keratoconus. Further work can be done with variations in the optimisation techniques and data augmentation techniques. Comparison of performance can be done by selecting reduced number of parameters, obtained from the measurements directly, with dimensionality reduction.

## Figures and Tables

**Figure 1:** Methodology flowchart.

**Figure 2:** Architecture of the CNN model used.

**Figure 3:** Performance metrics of CNN classification of PSO-optimised eye topography images.

**Figure 4:** Performance metrics of CNN classification of DPSO-optimised eye topography images.

**Figure 5:** Performance metrics of CNN classification of FPSO-optimised eye topography images.

**Table 1:** Machine learning techniques applied for keratoconus classification in the literature.

Authors	Classification	Network	Accuracy	Sensitivity	Specificity
Accardo et al.	Normal and keratoconus	BPN	98	93.3	98.6
Souza et al.	Normal and keratoconus	SVM	—	100	75
		MLP	—	100	75
		RBFNN	—	98	75
Toutounchian et al.	Normal, mild keratoconus, and keratoconus	MLP	77.6	—	—
		SVM	72	—	—
		DT	84	—	—
		RBFNN	71.2	—	—
Arbelaez et al.	Normal, abnormal, subclinical, and keratoconus	SVM	95.275	87.6	96.9
Hidalgo et al.	Astigmatism, forme fruste keratoconus, keratoconus, normal, and postrefractive surgery	SVM	88.8	77.22	97.02
Lavric et al.	Keratoconus, forme fruste keratoconus, and normal	QSVM	93	—	—
Santos et al.	Normal and keratoconus	CorneaNet	99.56		
Kamiya et al.	Normal and keratoconus 4 gradings	ResNet-18	99.1	100	98.4
Shi et al.	Normal, keratoconus, and subclinical	NN	93		
Kuo et al.	Normal and keratoconus	VGG16	93.1	91.7	94.4
		InceptionV3	93.1	91.7	94.4
		ResNet152	95.8	94.4	97.2
Lavric et al.	5 classes as normal, forme fruste, keratoconus II, keratoconus III, and keratoconus IV	SVM	AUC 0.88		
	3 classes as normal, forme fruste, and keratoconus	SVM	AUC 0.96		
	Normal and keratoconus	SVM	AUC 0.99		
Cao et al.	Normal and keratoconus	SVM	88.8		

**Table 2:** Confusion matrix and performance metrics of CNN classification of PSO-optimised eye topography images.

Actual classes	*N*	Predicted classes			Accuracy (%)	Specificity (%)	Sensitivity (%)
		Normal	Subclinical	Keratoconus			
Normal	492	464	19	9	93.8	96.7	89.1
Subclinical	424	41	364	19	93.3	93.9	91.7
Keratoconus	462	16	14	432	95.8	96.7	93.9

**Table 3:** Confusion matrix and performance metrics of CNN classification of DPSO-optimised eye topography images.

Actual classes	*N*	Predicted classes			Accuracy (%)	Specificity (%)	Sensitivity (%)
		Normal	Subclinical	Keratoconus			
Normal	492	472	16	4	95.0	97.7	90.6
Subclinical	424	35	372	17	94.3	94.7	93.5
Keratoconus	462	14	10	438	96.7	97.4	95.4

**Table 4:** Confusion matrix and performance metrics of CNN classification of FPSO-optimised eye topography images.

Actual classes	*N*	Predicted classes			Accuracy (%)	Specificity (%)	Sensitivity (%)
		Normal	Subclinical	Keratoconus			
Normal	492	476	12	4	95.4	98.1	90.8
Subclinical	424	36	376	12	95.1	95.1	94.9
Keratoconus	462	12	8	442	97.4	97.8	96.5

**Table 5:** Comparison of the proposed method with other machine learning approaches for detection and classification of keratoconus including forme fruste or mild cases of keratoconus.

Authors	Classification	Network	Accuracy
Proposed	Normal, mild keratoconus, and keratoconus	CNN	95.9
Toutounchian et al.	Normal, mild keratoconus, and keratoconus	MLP	77.6
		SVM	72
		DT	84
		RBFNN	71.2
Arbelaez et al.	Normal, abnormal, subclinical, and keratoconus	SVM	95.275
Hidalgo et al.	Astigmatism, forme fruste keratoconus, keratoconus, normal, and postrefractive surgery	SVM	88.8
Lavric et al.	Keratoconus, forme fruste keratoconus, and normal	QSVM	93
Kamiya et al.	Normal and keratoconus 4 gradings	ResNet-18	99.1
Shi et al.	Normal, keratoconus, and subclinical	NN	93

## Data Availability

The data used to support the findings of this study are included within the article.
